The article "Synthesis of Chitosan Microparticles Encapsulating Bacterial Cell-Free Supernatants and Indole Acetic Acid, and Their Effects on Germination and Seedling Growth in Tomato (Solanum lycopersicum)" was published in 2022. Journal: Int J Anal Chem.

# Synthesis of Chitosan Microparticles Encapsulating Bacterial Cell-Free Supernatants and Indole Acetic Acid, and Their Effects on Germination and Seedling Growth in Tomato (*Solanum lycopersicum*)

**DOI:** 10.1155/2022/2182783

**Published:** 2022-11-14

**Authors:** Thania Soledad Gonzalez-Montfort, Norma Almaraz-Abarca, Rocío Pérez-y-Terrón, Erik Ocaranza-Sánchez, Marlon Rojas-López

**Affiliations:** ^1^Instituto Politécnico Nacional, Centro De Investigación En Biotecnología Aplicada, Tepetitla, Tlax 90700, Mexico; ^2^Instituto Politecnico Nacional, Centro Interdisciplinario De Investigacion Para El Desarrollo Integral Regional, Unidad Durango, Sigma 119, Durango, Dgo 34220, Mexico; ^3^Benemerita Universidad Autonoma de Puebla, Facultad De Ciencias Biologicas, Puebla, Mexico

## Abstract

Encapsulation of biostimulant metabolites has gained popularity as it increases their shelf life and improves their absorption, being considered a good alternative for the manufacture of products that stimulate plant growth and fruit production. Cell-free supernatants (CFS) were obtained from nine indole-3-acetic acid (IAA) producing bacterial strains. *Stenotrophomonas maltophilia* (PT53T) produced the highest concentration of IAA (15.88 *μ*g/mL) after 48 h of incubation. CFS from this strain, as well as an IAA standard were separately encapsulated in chitosan microparticles (CS-MP) using the ionic gelation method. The CS-MP were analyzed by Fourier transform infrared spectroscopy (FTIR), showing absorption bands at 1641, 1547, and 1218 cm^−1^, associated with the vibrations of the carbonyl C=O, the N-H amine, and the bond between chitosan (CHI) and sodium tripolyphosphate (TPP). The effects of unencapsulated CFS, encapsulated CFS (EN-CFS), and encapsulated IAA standard (EN-IAA) on germination and growth of seven-day-old tomato (*Solanum lycopersicum*) seedlings were studied. Results showed that both EN-CFS and EN-IAA significantly (*p* < 0.05) increased seed germination rates by 77.5 and 80.8%, respectively. Both CFS and EN-IAA produced the greatest increase in aerial part length and fresh weight with respect to the treatment-free test. Therefore, it was concluded that the application of EN-CFS or EN-IAA could be a good option to improve the germination and growth of tomato seedlings.

## 1. Introduction

Plant growth-promoting bacteria (PGPB) or rhizobacteria (PGPR) establish mutualistic interactions with plants, promoting nutrient uptake, and water acquisition and help counteract the negative effects caused by biotic and abiotic stresses [1]. When applied to plants or the rhizosphere, substances produced by PGPB, known as phytohormones or biostimulants, interact with biochemical and physiological processes, influencing plant metabolism and morphology and promoting plant growth [1–5]. Several microorganisms can excrete phytohormones as secondary metabolites, depending on the composition of the medium and culture conditions. Indole-3-acetic acid (IAA), abscisic acid (ABA), gibberellin (GA), cytokinin, and ethylene are phytohormones that have physiological effects on plant development, affecting plant growth and promoting the induction of resistance systems against pathogens [6–8]. Phytohormones are considered biostimulants; these organic compounds are synthesized by all plants in certain organs and are transported to other tissues to perform their function[9]. At present, bacterial cell-free supernatants (CFS) containing biostimulants are an environmentally friendly alternative to the use of expensive agrochemicals, mainly because agrochemicals promote the accumulation of polluting compounds, increasing environmental pollution, decreasing the variability of microorganisms, and promoting soil degradation [10, 11].

Bacterial CFS is obtained by mechanical or physical separation of bacterial cells. Their composition includes substances from the culture medium, such as phytohormones and peptides, as well as microorganism biocontrol substances such as those obtained from *Bacillus* spp. (Iturin *A*, jasmonic acid, and surfactin, among others) [10]. Individual applications of these compounds have a positive effect on plants. Castiglione et al.[11] demonstrated that the combination of CFS with compost, algal extracts, humic acids, amino acids, or exopolysaccharides improved plant growth.

One of the most studied phytohormones is IAA, which belongs to the auxin group. IAA is a hydrophilic molecule with a structure similar to tryptophan, with an indole ring. IAA is involved in several physiological processes, such as cell differentiation and elongation, tissue differentiation, secondary and lateral root formation, and response to light and gravity [12–14]. Different bacterial genera synthesize IAA through different biosynthetic pathways, such as indole-3-pyruvate, indole-3-acetonitrile, indole-3-acetamide, tryptamine, side-chain tryptophan oxidase, and the tryptophan-independent pathway [15]. Bacterial synthesis of IAA may be associated with bacteria-plant interaction, as a colonization strategy benefited by phytostimulation. The most studied bacterial genera that produce IAA are *Azospirillum*, *Burkholderia*, *Erwinia*, *Enterobacter*, *Pseudomonas*, *Rhizobium*, *Serratia*, *Bacillus*, *Acinetobacter,* and *Sphingomonas* [4, 16].

Currently, microparticles containing bacterial phytohormones can be used as plant growth promoters, herbicides, fungicides, and pesticides. However, their size, as well as the use of toxic elements during their synthesis, may limit their use [17]. In contrast, chitosan encapsulates (CHI-ENC) have attracted attention, as chitosan (CHI) is a natural biomacromolecule and biopolymer formed by 2-acetamido-2-deoxy-*β*-1, 4-D-glucan chains. Chitosan (CHI) is mainly found in the exoskeletons of crustaceans and insects, as well as in the cell walls of some fungi, mainly Zygomycetes and algae [18–20]. The synthesis of CHI-ENC could help to keep biostimulant compounds stable, avoiding their rapid degradation and promoting a gradual release to plants or seeds. The most common method for CHI-ENC synthesis is ionic gelation, where the charge difference of the protonated amino groups of chitosan cross-links with the polyvalent tripolyphosphate anions (TPP) [19, 21].

CS-MP have a beneficial effect on plant seed germination, development, and growth, and helps to decrease the effects of abiotic stress, and increase resistance to diseases caused by pathogens due to their antimicrobial effects [22, 23]. Valderrama et al. [24], reported that chitosan nanoparticles (CS-NPs) loaded with IAA (mass ratio 1 : 0.25) applied to the lettuce variety *Crocantela* in hydroponic medium significantly improved both leaf length and dry weight. However, it was also observed that high concentrations of free IAA in the growth medium had a negative effect on root length. Hoang et al. [25] reported the potential use of CS-NPs alone on root length, showing increases between 7.1 and 71%, depending on concentration, encapsulated metabolites, and plant species. In plants such as coffee, corn, wheat, chicken, and tomato, it has been observed that this type of encapsulation has had a good effects on the length of the aerial part, fresh and dry weight, total chlorophyll, germination, number of leaves, leaf area, stem diameter, vigor index, the number of secondary roots, as well as protection against certain pathogens such as *F. oxysporum*, *C. gloeosporioides*, *P. capsici*, *S. sclerotium*, *G. fujikuori*, *A. solani*, *F. graminearum*, and *C. michiganensis*.

The aim of the present study was to synthesize chitosan microparticles containing bacterial CFS with IAA. Once obtained, the effect of their application on the germination and growth of tomato seedlings were evaluated.

## 2. Materials and Methods

### 2.1. Inoculum Preparation

Table 1 shows the IAA-producing bacterial strains used in the present study. Six strains were obtained from the bacterial collection of the Facultad de Ciencias Biológicas-Benemérita Universidad Autónoma de Puebla (FCB-BUAP), Mexico, after identification by the same institution using the API20NE test. Three strains were obtained from the bacterial collection of the Centro de Investigación en Biotecnología Aplicada-Instituto Politécnico Nacional (CIBA-IPN), Mexico, and identified using a molecular test (16S gene). The strains were grown in nutrient broth (BD Bioxon, 8 g/L) at 32°C with continuous agitation at 120 rpm for 24 h for CFS production.

### 2.2. Quantitative Determination of IAA in Bacterial Culture Media

Bacterial populations obtained after 24 h were adjusted to 10^8^ cfu/mL, and 1 mL of each solution was inoculated into 25 mL of nutrient broth supplemented with 0.5 g/L L-tryptophan (L-trp) (Meyer) at pH 7 [7]. Culture conditions were maintained at 32°C and 120 rpm for 48, 72, and 96 h to evaluate IAA production as a function of time. After this time, the growth medium was centrifuged at 4709 × *g* for 15 min at 4°C and the CFS was obtained. 500 *μ*L of this suspension was added to 500 *μ*l of Salkowski reagent (2 mL 2.5 M FeCl_3_ + 50 mL HClO_4_ 50% (v/v)), and the well-integrated mixture was incubated at room temperature for 30 min. Absorbance at 535 nm [26, 27] was determined to correlate with IAA concentration using a standard curve in the range of 2–100 *μ*g/mL. PT53T was the strain with the highest IAA production, as was subsequently corroborated by FTIR analysis (Bruker Vertex 70; spectral range of 4000–400 cm^−1^ using 120 scans, in mode attenuated total reflectance (ATR) sampling cell for analysis).

### 2.3. CFS Lyophilization

Bacterial cells were removed from the growth medium by centrifugation at 7358 × *g* for 20 min to obtain the supernatant. Then, supernatants were frozen at 20°C for 24 h, followed by ultrafreezing at −80°C for 5 days, and finally, lyophilized (Labconco, Mod. FreeZone 1L Freeze Dry System) at 51°C and 0.054 mbar to obtain CFS.

### 2.4. Preparation of Chitosan Encapsulates

Chitosan microparticles (CS-MP) were prepared by the ionic gelation method proposed by Antoniou et al. [28], with some modifications. Medium molecular weight chitosan (CHI, 75%–85% deacetylate, Sigma–Aldrich, 448877) was dissolved at a concentration of 0.5 mg/mL in a 1% v/v aqueous solution of acetic acid (Meyer CAS: 64-19-7). Four different pH values (4, 4.5, 5, and 5.5) were studied by adjusting the solution with 10 M NaOH (Meyer CAS 1310-73-2). A solution of sodium tripolyphosphate (TPP; Meyer CAT 7005–500g) 0.7 mg/ml was added dropwise to the chitosan solution in a 3 : 1 ratio with vigorous magnetic stirring at room temperature. CFS and IAA standard (98%, Sigma–Aldrich, I3750) at concentrations of 15.88, 158.88, 1588, and 15880 *μ*g/mL were encapsulated at pH 5, to be subsequently used for inoculation of tomato seeds. All samples were prepared in triplicates and centrifuged at 11337 × *g* for 30 min at room temperature. The supernatant was used for UV-vis measurements, and the precipitate was allowed to dry for analysis by FTIR spectroscopy.

### 2.5. Morphology and Particle Size

Morphology and size of the CS-MP were observed using a SEM-FE-JOL 7610F scanning electron microscope (Tokyo, Japan) with Oxford EBSD detector with 2.0 kV voltage accelerations and secondary electron detector (SEI). Samples of CS-MP were dry mounted on carbon tape and were coated with Au/Pd. The SEM images obtained were analyzed with ImageJ 1.52a software (National Institute of Health, USA) to determine the average particle size.

### 2.6. Fourier Transform Infrared Spectroscopy (FTIR)

CS-MP containing bacterial CFS (EN-CFS) and standard IAA (EN-IAA) were analyzed using a Bruker Vertex 70 Fourier transform infrared spectrometer in the spectral range of 4000–400 cm^−1^ using 120 scans. CS-MP samples were placed on the surface of the attenuated total reflectance (ATR) sampling cell for analysis.

### 2.7. Determination of the Encapsulation Efficiency

Suspensions with EN-CFS and EN-IAA were centrifuged at 11337 × *g* for 30 min. The supernatant was separated for analysis by UV-VIS spectrophotometry. The amount of IAA present in the supernatant was estimated using an IAA calibration curve. Similarly, the encapsulation efficiency of EN-IAA was determined as a function of the IAA present in the supernatant using equation (1) [29], where IAA_i_ is the initial amount of IAA and IAA_s_ is the amount in the supernatant.

(1) $$\begin{array}{c} \text{Encapsulation}\%=\left(\frac{\text{IAA}i-\text{IAA}s}{\text{IAA}i}\right)*100. \end{array}$$

### 2.8. Inoculation of CS-MP in Tomato Seeds

The tomato (*Lycopersicum esculentum;* ball-type) seeds were obtained from the brand Hortaflor. For inoculation with CFS, EN-CFS, and EN-IAA the first three rinses were performed with sterile distilled water, then, they were disinfected using 70% alcohol for 10 min and rinsed with sterile distilled water five times [30]. *In vitro,* forty seeds were inoculated with 1 mg/mL of encapsulate, placed on 60% agar, and left to develop for 7 days at 30°C in darkness [31]. The germination rate, root length, and aerial part length (Steren vernier mod. HER-411) as well as fresh weight (American Weigh GEMINI-20 Portable Milligram Scale) of 25 seedlings was recorded.

### 2.9. Experiment Design and Statistical Analysis

The experiment consisted of two factors: (*A*) metabolite concentration, and (*B*) type of metabolite presentation (or method for its preparation). Four experimental variables were studied after 7 days of seedling growth: germination rate, root length, aerial part length, and fresh weight. Factor *A* included five levels of metabolite concentration (0, 15.88, 158.8, 1588, and 15880 *μ*g/mL) which were adjusted according to their order of magnitude, using the IAA obtained from strain PT53T as the reference and considering sterile distilled water as the negative control (zero). Factor B included three levels: CFS, EN-ECFS, and EN-IAA. All experiments were performed in triplicate and were analyzed with the Kolmogorov–Smirnov normality test using Statistica v14.0.0.15 software. The results shown in the figures are expressed as mean ± standard deviation (SD). The significance level of the variation between treatments was evaluated using a two-way analysis of variance (ANOVA). The mean values were separated using the Tukey's test (*p* < 0.05). Response surface analysis was performed using MINITAB16 and Excel software.

## 3. Results and Discussion

### 3.1. Production of Bacterial CFS Containing IAA

All strains evaluated showed IAA production, with *Stenotrophomonas maltophilia* (PT53T) being the strain that produced the highest concentration of IAA after 48 h of culture. On the other hand, *Ewingella americana* (S17) and *Brevundimonas vesicularis* (2H2B) showed the highest production at 72 and 96 h, respectively (Table 2). Based on these results, strain PT53T was selected for further studies.

Production of IAA as a bacterial secondary metabolite is affected by pH value, temperature, culture medium composition (carbon and nitrogen source), bacterial species, growth stage (stationary phase), and the addition of different concentrations of L-trp [30, 32–34]. It has been shown that *S. maltophilia* can promote plant growth, stimulate pathogen control, and increase plant tolerance to different types of stresses due to the production of phytohormones such as IAA and protective enzymes [35]. Adeleke et al. [36] demonstrated that genes such as *trp*ABCD, *ami*E, and *mia*A present in this bacterium were related to IAA synthesis through the indole-3-acetamine pathway.

The concentration of IAA produced by the *S. maltophilia* strain is considered low. However, the addition of different concentrations of L-trp contributed significantly to the increase in IAA production, ranging from 3.9 *μ*g/mL to 2.5 mg/mL [30, 32–34, 36]. Growth of the bacterium in LB medium spiked with L-trp as a precursor at a concentration of 25 ug/mL produced a 24% increase in IAA within 24 h. It was also observed that higher concentrations (100–400 ug/mL) of the precursor increased IAA production to 79 ± 2. 55 ug/mL. However, studies carried out over a longer period (7 days) reported concentrations of 30 ug/mL [37]. Yeast malt dextrose (YMD) medium supplemented with 0.1% L-trp and an incubation time of 4 days resulted in an IAA concentration of 2.5 mg/mL in the medium for *S. maltophilia* BE25 isolated from the roots of banana [30]. In contrast, a decrease in IAA production was observed for longer incubation periods [38].

FTIR analysis for the IAA standard (Figure 1 (1), the nutrient broth (control) (Figure 1 (2)) and the extracts (Figures 1, (3–5), corresponding to the 3 strains with the highest IAA production (PT53T, S17, and 2H2B) are shown in Figure 1. Absorption bands at 1636 cm^−1^ show the -C=O stretching vibration of the carboxylic group. The peaks centred between 1350–1650 cm^−1^ arise from the asymmetric alkyl (-CH2) stretching group, and the peak at 1094 cm^−1^ is related to the C-H bending vibration [39–41].

### 3.2. UV-VIS Spectrophotometric Analysis

Maximum intensity for all spectra was obtained at 280 nm (Figure 2), from the lowest to the highest concentration of IAA (24–85 *μ*g/mL). The calibration equation for the IAA standard (*y* = 0.029*x* + 0.121) was obtained from a linear relationship between the maximum intensity of the band at 280 nm and a known concentration of IAA. The readings correspond to the presence of IAA in the supernatant [42, 43].

Figure 3 shows the UV-VIS absorbance values at 280 nm of the IAA standard measured in the supernatant after centrifugation (left axis) once the encapsulation of the IAA standard was performed by applying the two types of initial reactions TPP + IAA and CHI + IAA respectively. The encapsulation efficiency (right axis) of chitosan particles was estimated from the IAA concentration in the supernatant using the calibration equation and, subsequently, equation (1).  Table 3 shows both the IAA concentration determined in the supernatant and the encapsulation efficiency. For pH 4 and 4.5 the suspension was transparent; however, for pH 5 and 5.5, the suspension was opalescent. The highest encapsulation efficiency (85.88%) was observed at pH 5, when IAA was added to TPP (initial reaction TPP + IAA).

From UV-VIS spectrophotometry measurements, it was found that when IAA was added to CHI (during the CS-MP preparation procedure), the amount of free IAA was high in the supernatant and the encapsulation efficiency was low. However, when IAA was incorporated into TPP, the concentration of free IAA in the supernatant was low (20–35 *μ*g/mL) and the encapsulation efficiency was high (80%–85%). Similarly, when both IAA and bacterial CFS were added to chitosan, a low percentage of encapsulation was obtained, being at pH 5.5, the condition that presented the highest percentage of encapsulation (54.74%).

### 3.3. FTIR Analysis of EN-CFS and EN-IAA

When TPP was incorporated into chitosan (CHI) during encapsulation of the IAA standard and CFS, the translucent solution became opalescent, suggesting an electrostatic interaction between chitosan and TPP; Agarwal et al. [21], mentioned that this effect corresponded to the formation of small particles. At pH 4, 5 and 5.5, a higher opalescence was observed for both control particles (blank particles) and those containing the standard IAA or CFS. The opalescence is related to both TPP-CHI interaction and pH, although at pH below 4.5 particles synthesis is unlikely. However, at pH levels above 5, more homogeneous suspensions are generated [44].

Figure 4 shows the FTIR spectra of both the precursors (CHI and TPP) and the particles obtained and used to encapsulate the standard IAA and the CFS. The spectrum of chitosan shows two absorption bands at 1154 and 1075 cm^−1^, which are related to the asymmetric C-O-C stretching of the glycosidic bond and C-O stretching vibrations, respectively [21]. The spectrum of TPP shows two bands at 1210 cm^−1^ and 899 cm^−1^, which may be associated with P=O stretching and P-O/P-O-P vibrations, respectively [45, 46]. When both compounds (CHI and TPP) react to form target particles, the resulting FTIR spectra show three specific bands that result from their interaction. These bands were observed at 1641, 1547, and 1218 cm^−1^; and are associated with the carbonyl C=O, the N-H amine, and the bond between CHI and TPP, respectively, indicating particle formation [47, 48].

The FTIR spectra of the EN-CFS and EN-IAA showed the same three absorption bands at 1642, 1547, and 1218 cm^−1^, as shown in Figure 5, related to the formation of CS-MP. No other bands corresponding to CFS metabolites were observed, suggesting that CFS was inside the microparticles, as indicated by the UV-VIS results. In addition, other absorption bands were observed at 1450 and 1690 cm^−1^ corresponding to alkyl (-CH_2_) and carbonyl, respectively. All these results agree with those reported by Sachdev et al. [32] and Patel and Patel [40].

### 3.4. Morphology and Size of Microparticles

Morphology and particle size of CS-MP were analyzed by scanning electron microscopy. In the case of the encapsulated control (blank CS-MP), their size was 2.31 ± 0.86 *μ*m (Figure 6(a)), achieving larger sizes than those reported by Antoniou et al. [28]. However, this difference could arise from the molecular weight (100 kDa) and degree of deacetylation (90%) used by those researchers in contrast to the parameters used in this research (190–310 kDa, 75%–85%). The shape and size of microparticles are affected by the pH, the molecular weight of chitosan, the concentration of the solutions, the CHI/TPP molecular ratio, as well as the agitation conditions and the percentage of acetic acid used [49, 50]. For EN-CFS at concentrations of 15.88 and 15880 *μ*g/mL, an average particle size of 7 ± 1.95 and 2.76 ± 0.160 *μ*m, respectively, was determined (Figures 6(b) and 6(c)). EN-IAA containing 15.88 and 166 *μ*g/mL of the IAA standard showed average sizes of 3.98 ± 0.160 *μ*m (Figure 6(d)) and 4.65 ± 0.076 *μ*m (Figure 6(e)), respectively. Several studies have shown that the increase in particle size is a consequence of IAA addition and effective encapsulation of this metabolite [24, 51]. In addition, several clusters were observed, possibly related to a flocculation effect by the interaction of the charges because of the addition of the positive charge of IAA [52]. Several reports mention that in a 3 : 1 ratio (CHI: TPP) there is the possibility of aggregate formation [21].

### 3.5. Tomato Seed Inoculation and Seedling Growth

Figure 7 shows the results for the variables considered in the experimental design: germination rate, root length, aerial part length, and fresh weight. Results were obtained after seedlings were allowed to grow for 7 days (Figure 8).

All four variables: germination rate, root length, aerial part length, and fresh weight were influenced by the two factors previously defined, as was shown by a two-way ANOVA analysis.  Table 4 summarizes the main statistical parameters commonly used to determine whether a treatment can affect a set of specific variables (responses).

Figure 9 shows the response surface and contour plots of the combined effect of both factors (metabolite concentration and method) on germination rate and root length, respectively. According to the germination rate response surface and contour plot, a metabolite concentration of 15.88 at 15880 *μ*g/mL using method 2 (EN-CFS) generates a germination rate of 80.8% (Figures 9(a) and 9(b). A similar result of 77.5%, was achieved with method 3 (EN-IAA) using 15.88 *μ*g/mL, and finally, a germination rate of 80% was achieved with method 1(CFS) at 158.8 *μ*g/mL metabolite concentration. For the root length response surface and contour plot, a decrease in root length was observed for all metabolite concentrations (Figures 9(c) and 9(d) although a slight increase was observed for a concentration of 15.88 mg/mL using method 2. Figures 10(a)–10(d) shows the response surface and contour plots of the combined effect of both factors (metabolite concentration and method) on aerial part length and fresh weight, respectively. According to the response surface of aerial part length and contour plot, the optimum value of 8.27 cm was obtained using method 3 (encapsulated IAA standard) at 15.88 *μ*g/mL (Figures 10(a) and 10(b)). Finally, for the fresh weight response surface and contour plot, an optimum value of 0.04 g was obtained using method 1 (free bacterial SFC) (Figures 10(c) and 10(d)). Another optimum value of 0.04 g was also obtained using method 3 (the encapsulated IAA standard) at 15.88 *μ*g/mL.

Rapid degradation of IAA and CFS is one of the disadvantages of their exogenous application, which is increased by several factors such as salinity, temperature, and the use of agrochemicals [10]. However, microencapsulation of these metabolites has shown enhanced absorption efficiency with beneficial effects on plants [53]. In this research, EN-CFS (method 2) and EN-IAA (method 3) were the best alternatives to improving germination rate (Figures 7(a) and 7(b)). Currently, different strategies have been studied, such as those applied in this research to enhance plant growth. The use of PGPR, biostimulants, and recently the implementation of chitosan-based encapsulants have been studied, the final products being applied either via foliar or on plant roots. Different authors have pointed out that the addition of chitosan encapsulates or their derivatives has shown a positive effect on the increase in biomass, root length, flowering, mycorrhization, biocontrol, and even on the increase in phytohormone production [31, 32, 54, 55].

In tomato seeds, inoculation with 0.1 mg/mL of empty CS-NPs had a positive effect on germination percentage, fresh and dry weight, length, and vigour of seedlings. In addition, results showed that these particles induced plant defence response as well as the production of salicylic acid (SA), jasmonic acid (JA), abscisic acid (ABA), and the activation of metabolic pathways involved with the biosynthesis of phenolic compounds [31, 55, 56]. Andrade et al. [57] used chitosan-alginate nanoparticles loaded with IAA and bacterial IAA, adding them to plants 25, 30, and 45 days after transplanting, and observed a significant effect on plant growth. In other plants, such as wheat, the addition of CS-NPs at concentrations of 5 *μ*g mL^−1^ to seeds generated a positive effect on germination and seedling length, as well as an increase in the number of adventitious roots [23]. Comparing our results with those reported in the mentioned literature, our encapsulated products showed a good effect on tomato seed germination and seedling growth. However, when increasing the concentration of IAA, a decrease in root and aerial part length was observed. This agrees with other reports in the literature that point out that low auxin concentrations have a stimulatory effect on plant growth, while higher auxin concentrations have an inhibitory effect [30, 40, 58].

## 4. Conclusions

The use of bacterial CFS containing biostimulant compounds such as IAA and its form in chitosan microparticles could represent a good option for germination and seedling growth. In addition, these particles reduce their sensitivity to light, humidity, temperature, and soil components, increasing their shelf life and minimizing their exposure to contamination during the application process. Thus, CFS and EN-CFS would avoid the use and release of bacteria into the environment, especially because approximately 10^8^–10^9^ CFU/g are needed to have a successful commercial product for crop improvement, in addition, some authors suggest checking the toxin production or pathogenicity of the strains used. In the future, biofertilizers, including CFS encapsulated in chitosan could generate a crucial change in the development of sustainable approaches to crop production. Experimental studies at other stages of tomato development and in other plant species could be necessary to find other forms of application to understand the mechanism of interaction between the plant and the microparticles, as well as to observe the process of metabolite release once the encapsulates are opened.

## Figures and Tables

**Figure 1:** FTIR spectra of the bacterial CFS: (1) IAA standard, (2) nutritive broth control, (3) 2H2B, (4) S17, and (5) PT53T.

**Figure 2:** UV-VIS spectrum of the IAA standard at several concentrations.

**Figure 3:** UV-VIS absorbance of the IAA standard at 280 nm measured in the supernatant (left axis) and, the encapsulation efficiency as a function of the concentration of IAA (right axis).

**Figure 4:** FTIR spectra of the precursors CHI (purple) and TPP (blue) and, also of the CS-MP control (black) obtained from the interaction of both compounds.

**Figure 5:** FTIR spectra of EN-CFS, EN-IAA, and CS-MP control.

**Figure 6:** Scanning electron microscopy images of CS-MP blank particles (a), EN-CFS at 15.88 *μ*g/mL (b), and 15880 *μ*g/mL (c), EN-IAA at 15.88 *μ*g/mL (d), and 166 *μ*g/mL (e).

**Figure 7:** Experimental data obtained for the responses selected for this design of experiment: (a) germination rate, (b) root length, (c) aerial part length and, and (d) fresh weight. Bacterial CFS, EN-CFS, and EN-IAA. 95% Tukey's simultaneous confidence intervals, means that do not share a letter are significantly different; capital letters: concentration factor, lower case letters: application mode factor.

**Figure 8:** Effect of CS-MP on tomato root and aerial part length seedling; method: (a) CFS, (b) EN-CFS, and (c) EN-IAA, metabolite concentration (*μ*g/mL): (A) 15.88 (B) 158.8, and (C) 1588, (D).

**Figure 9:** Response surface and contour plots determined for the germination rate, root length: method: (1) CFS, (2) EN-CFS, and (3) EN-IAA; metabolite concentration (*μ*g/mL): (0) water, (1) 15.88, (2) 158.8, (3) 1588, and (4) 15880 *μ*g/mL.

**Figure 10:** Response surface and contour plots determined for the aerial part length and fresh weight: (1) CFS, (2) EN-CFS, and (3) EN-IAA. Metabolite concentration (*μ*g/mL): (0) water, (1) 15.88, (2) 158.8, (3) 1588, and (4) 15880.

**Table 1:** Indole acetic acid producing bacterial strains used in the study.

Number	Code of strains	Source of bacterial isolate	Species	Collection	Identification method (%)	
					API20NE	Molecular (16S gene)
**1**	2S3BA	Rhizosphere of tomato plant	*Stenotrophomonas maltophilia*	FCB-BUAP	73.4	
**2**	1S4AA	Rhizosphere of tomato plant	*Chryseobacterium indologenes*	FCB-BUAP	86.2	
**3**	2S1A	Rhizosphere of tomato plant	*Sphingomonas paucimobilis*	FCB-BUAP	98.7	
**4**	2S1C	Rhizosphere of tomato plant	*Chromobacterium violaceum*	FCB-BUAP	93.3	
**5**	TH3A	Tomato plant leaf	*Burkholderia cepacia*	FCB-BUAP	97.7	
**6**	2H2B	Tomato plant leaf	*Brevundimonas vesicularis*	FCB-BUAP	99.3	
**7**	S17	CIBA soil	*Ewingella americana*	CIBA-IPN		99.9
**8**	MT11PS	Rhizosphere of potato plant	*Leclercia adecarboxylata*	CIBA-IPN		99.7
**9**	PT53T	Rhizosphere of potato plant	*Stenotrophomonas maltophilia*	CIBA-IPN		99.6

FCB-BUAP: Facultad de Ciencias Biológicas-Benemérita Universidad Autónoma de Puebla, Mexico. CIBA-IPN: Centro de Investigación en Biotecnología Aplicada-Instituto Politécnico Nacional, Mexico.

**Table 2:** Indole acetic acid (IAA) production (*μ*g/mL) by nine bacterial strains after incubation periods.

Incubation time (h)	Strains								
	2S3BA	2S1C	2S1A	2H2B	TH3A	1S4AA	PT53T	S17	MT11PS
48	4.601	4.932	7.033	3.723	5.599	1.247^*∗*^	15.880^*∗∗*^	7.093	4.691
72	9.634	7.828	7.566	8.683	6.537	8.278	5.059^*∗*^	12.691^*∗∗*^	7.273
96	6.757	10.058	9.216	10.104^*∗∗*^	7.993	4.241	2.920^*∗*^	9.839	6.357

^*∗*^Lower IAA production; ^*∗∗*^high IAA production. Bacterial strains according to Table 1.

**Table 3:** Effect of pH on the chitosan particle formation.

Encapsulation treatment	pH	IAA concentration supernatant (*μ*g/mL)	Encapsulation (%)
Control	4.0	0	100
Control	4.5	0	100
Control	5	0	100
Control	5.5	0	100

CHI + IAA	4.0	81.91	48.24
CHI + IAA	4.5	83.79	51.86
CHI + IAA	5	82.61	53.13
CHI + IAA	5.5	84.86	54.74

TPP + IAA	4.0	30.89	80.73
TPP + IAA	4.5	26.13	85.37
TPP + IAA	5	24.48	85.88
TPP + IAA	5.5	28.30	80.03

CHI + IAA: IAA added to chitosan; CHI + TPP: TPP added to chitosan.

**Table 4:** Two-way ANOVA analysis for the statistical comparison of features studied in tomato seedlings.

	Source of variation	Sum of squares	Degree of freedom	Mean square	*F* value	*p* value
Germination rate	Concentration	963.69	5	192.74	3.67	0.0088
	Method	1085.37	2	542.68	10.32	0.0003
	Interaction	1268.76	10	126.88	2.41	0.0258

Root length	Concentration	355.69	5	71.14	87.04	3.68 *E* − 63
	Method	9.49	2	4.74	5.81	3.25 *E* − 03
	Interaction	58.41	10	5.84	7.15	1.88 *E* − 10

Aerial part length	Concentration	355.69	5	71.14	87.04	3.68 *E* − 63
	Method	9.49	2	4.74	5.81	3.25 *E* − 03
	Interaction	58.41	10	5.84	7.15	1.88 *E* − 10

Fresh weight	Concentration	0.0002	5	3.6 *E* − 05	0.32	0.902147
	Method	0.0027	2	1.3 *E* − 03	11.80	0.000010
	Interaction	0.0041	10	4.1 *E* − 04	3.61	0.000127

## Data Availability

The (https://1drv.ms/u/s!AheVVJ1zvLUX8z7zx8zw7zmU3zAH?e=ATpnkq) data used to support the findings of this study are included within the article.
